# Edible Bird's Nest Regulates Hepatic Cholesterol Metabolism through Transcriptional Regulation of Cholesterol Related Genes

**DOI:** 10.1155/2022/8882993

**Published:** 2022-06-09

**Authors:** Zhang Yida, Hussah Al-Shuwayah, Maznah Ismail, Mustapha Umar Imam

**Affiliations:** ^1^Cardiology Department, Kangjixintu Hospital, Hebei, China; ^2^Department of Biology, College of Science, Imam Abdulrahman Bin Faisal University (IAU), Dammam 31441-1982, Saudi Arabia; ^3^Laboratory of Molecular Biomedicine, Institute of Bioscience, Universiti Putra Malaysia, 43400 Serdang, Selangor, Malaysia; ^4^Department of Medical Biochemistry, Faculty of Basic Medical Sciences, College of Health Sciences, Usmanu Danfodiyo University, Sokoto, Nigeria; ^5^Centre for Advanced Medical Research and Training, Usmanu Danfodiyo University, Sokoto, Nigeria

## Abstract

**Objective:**

Hypercholesterolemia is a strong risk factor for cardiovascular diseases. Side effects associated with the use of pharmaceutical agents can cancel out their benefits. Dietary management of hypercholesterolemia is, therefore, receiving much attention due to fewer side effects. In this study, we explored the effectiveness of edible bird's nest (EBN) in the prevention of hypercholesterolemia in rats.

**Methods:**

High-cholesterol diet (HCD) (4.5% cholesterol and 0.5% cholic acid) with or without EBN (low (2.5%) or high dose (20%)) was given to rats for 12 weeks, and their weights were observed. Simvastatin (10 mg/kg/day) was administered for the same period as a control drug. Serum and tissue samples were collected at the end of the study, from which biochemical parameters (lipid profiles, oxLDL, liver enzymes, urea, creatinine, uric acid, and lipase activity) and hepatic mRNA levels were measured.

**Results:**

The HCD group had higher levels of serum lipids, liver enzymes, uric acid, urea, and lipase activity compared with those of the other groups. The hepatic mRNA levels of cholesterol metabolism genes (APOB, PCSK9, HMGCR, LDLR, and CYP7A1) in the HCD group also tended toward increased cholesterol production and reduced cholesterol clearance. EBN, especially the highest dose, attenuated the HCD-induced changes, partly through improving the transcriptional regulation of hepatic cholesterol metabolism genes with fold changes of 0.7, 0.6, 0.5, 1.7, and 2.7, respectively, in comparison to the HCD group. In fact, EBN produced better results than simvastatin.

**Conclusion:**

Thus, the results suggest that EBN can regulate cholesterol metabolism and, therefore, be a source of functional ingredients for the management of hypercholesterolemia.

## 1. Introduction

Hypercholesterolemia is a common metabolic problem that is implicated in the development of cardiovascular diseases (CVD) [1]. Genetic predisposition can be the basis of hypercholesterolemia, although the majority of metabolic perturbations leading to hypercholesterolemia result from lifestyle factors. Accordingly, dietary choices and level of physical activity are strong determinants of the levels of lipids in the blood of individuals [2]. In addition to CVD, hypercholesterolemia tends to develop in patients with other metabolic diseases like type 2 diabetes and metabolic syndrome [3]. Clinical diagnosis of hypercholesterolemia is performed using the lipid profile levels, in which case elevated serum total cholesterol (TC), low-density lipoprotein and triglycerides, and decreased serum high-density lipoprotein have been associated with the development of clinical disease and poor outcomes if not managed appropriately.

Lipid-lowering drugs have been used to control the risk of diseases caused by hypercholesterolemia, although success has been limited due to side effects or lack of efficacy [4]. What makes clinical management particularly challenging is the underlying metabolic perturbations leading up to overt hypercholesterolemia. Transcriptional changes in several cholesterol metabolism genes have been shown to underlie the changes in lipid profiles, and as such, effective management of hypercholesterolemia should not only entail the biochemical regulation of serum lipids but also the regulation of lipid-producing machinery. The pharmaceutical agents that target a single biochemical process are limited in their efficacy due to this challenge, and in recent years, dietary management has received attention with a view to targeting multiple biochemical and possibly transcriptional mechanisms that underlie hypercholesterolemia. Thus, foods with multiple bioactive compounds have been proposed for managing diseases with multiple metabolic perturbations [5, 6].

Edible bird's nest (EBN) is produced by swiftlets and has been consumed for over a thousand years in China. It is increasingly becoming a famous nutraceutical in Asia as a result of its health-promoting effects. Although it has been used in the past, based on traditional belief, scientific evidence is now providing an explanation for its efficacy [7]. We have previously demonstrated the anti-inflammatory, antioxidative, anticoagulant, and antihyperglycemic effects of EBN in high-cholesterol diet-fed rats [8–10]. In the present study, we show that EBN is also able to prevent hypercholesterolemia in HFD-fed rats through the regulation of hepatic cholesterol metabolism.

## 2. Materials and Methods

### 2.1. Materials

EBN was purchased from Blossom View Sdn. Bhd (Terrengganu, Malaysia) while simvastatin was purchased from Hangzhou MSD Pharmaceutical Co., Ltd (Hangzhou, China). Standard rat pellets were purchased from Specialty Feeds (Glen Forrest, WA, USA), cholesterol was purchased from Amresco (Solon, OH, USA), cholic acid was purchased from Santa Cruz Biotechnology (Santa Cruz, CA, USA), and palm oil was purchased from Yee Lee Edible Oils Sdn. Bhd. (Perak, Malaysia). Analytical grade ethanol was purchased from Merck (Darmstadt, Germany), while RCL2 solution was purchased from ALPHELYS (Toulouse, France). Lipid profile kits were purchased from Randox Laboratories Ltd. (Crumlin, County Antrim, UK), while an oxLDL ELISA kit was purchased from Elabscience Biotechnology Co., Ltd (Wuhan, China). An RNA extraction kit was purchased from RBC Bioscience Corp. (Taipei, Taiwan), and a GenomeLab™ GeXP Start Kit was purchased from Beckman Coulter Inc (Miami, FL, USA).

### 2.2. Animal Handling and Feeding

In this study, we followed the methods of Hou et al. [11]. Similarly, we have previously reported the compositional analysis of the EBN sample used in this study [8]. Accordingly, the ethical permission for the animal study was given by the Animal Care and Use Committee (ACUC) of the Faculty of Medicine and Health Sciences, Universiti Putra Malaysia (Project approval number: UPM/IACUC/AUP-R011/2014). Thirty Sprague-Dawley rats (10 weeks old, 230–280 g) were handled as stipulated by standard guidelines for handling animals. The rats were housed at 25 ± 2°C, 12/12 h light/dark cycle and allowed to acclimatize for 2 weeks with free access to normal pellets and water. The rats were then divided into 5 groups: the normal group fed with normal pellet; the HFD group fed with HFD containing 4.5% cholesterol and 0.5% cholic acid; the HFD + SIM group fed with HFD and simvastatin (10 mg/kg/day); and 2 EBN groups fed with low- (2.5%) or high-dose (20%) EBN and HFD. The intervention lasted 12 weeks, and body weights were measured weekly while food intake was calculated every day by subtracting the leftover from what was added the previous day. Rats were sacrificed at the end, and their blood and tissue samples were collected for further analyses.

### 2.3. Biochemical Analyses

Serum samples were analyzed for lipid profile (TC, LDL, HDL, and triglyceride), liver enzymes (ALT, AST, and ALP), LDH, urea, creatinine, uric acid, and lipase activity using Randox analytical kits on Selectra XL instrument (Vita Scientific, Dieren, the Netherlands).

### 2.4. Serum Oxidized LDL

Serum oxidized LDL was analyzed using an oxLDL ELISA kit according to the manufacturer's recommendations. Absorbances were read using a BioTeK Synergy H1 Hybrid Reader (BioTek Instruments Inc., Winooski, VT, USA) at the recommended wavelength (450 nm), and results were analyzed on https://www.myassays.com using linear regression (*R*^2^ = 0.9989, *y* = 0.1258x − 0.0041).

### 2.5. Histology

Liver samples were fixed in 10% formalin and used for histological evaluation using an automated tissue processor (Leica TP 1020). Slides were then stained with haematoxylin and eosin, and examined under a standard light microscope.

### 2.6. Gene Expression

#### 2.6.1. Primer Design

The primers used in this study were designed with the GenomeLab eXpress Profiler software using input sequences from the National Center for Biotechnology Information website (https://www.ncbi.nlm.nih.gov/nucleotide/). The primers were tagged with an 18-nucleotide universal forward and a 19-nucleotide universal reverse sequence, respectively (Table 1). They were synthesized by Integrated DNA Technologies (Singapore).

#### 2.6.2. RNA Extraction, Reverse Transcription, and PCR

RNA was extracted using an RNA isolation kit (RBC Biotech Corp., Taipei, Taiwan) and diluted to 20 ng/mL. Reverse transcription and PCR programs were performed according to the GenomeLab™ GeXP Start Kit protocol (Beckman Coulter, USA), as shown in Table 1.

#### 2.6.3. GeXP Genetic Analysis System and Multiplex Data Analysis

A sample loading solution (38.5 *μ*L) and DNA size standard 400 (0.5 *μ*L) (GenomeLab GeXP Start Kit; Beckman Coulter, Inc, USA) were mixed with 1 *μ*L PCR products, and the mixture was loaded onto a 96-well sample plate for analysis on the GeXP genomelab genetic analysis system (Beckman Coulter, Inc, Miami, FL, USA). Gene expression results were analyzed with the Fragment Analysis module of the GeXP system software to get the real peak for the corresponding gene, and the data were exported and normalized on eXpress Profiler software [10].

### 2.7. Data Analysis

Data are presented as a mean ± standard deviation. A normality test was conducted to confirm normal distribution, and comparisons of the means were performed using a one-way analysis of variance (ANOVA) on SPSS 17.0 software (SPSS Inc., Chicago, IL, USA). The significance of the difference between the comparisons was determined by Tukey's range test. *p* < 0.05 was considered significantly different.

## 3. Results and Discussion

### 3.1. Food Intake and Body Weight

Table 2 shows that the food intake (calories) of the different groups during the intervention period was similar. Similarly, the body weights after 12 weeks are shown in Table 2. No significant differences were observed between the groups after 12 weeks of intervention although the percentage body weight changes were different. The HFD, HFD + SIM, HFD + EBNL, and HFD + EBNH groups had 50%, 40%, 45%, and 43% changes in body weights, respectively.

### 3.2. Lipid Profile

Table 2 also shows the lipid profiles of the different groups. The normal group had a significantly lower cholesterol level than the other groups. The cholesterol levels of the EBN groups were lower than those of the HFD group, although it was only significantly so for the HFD + EBNH group (*p* < 0.05), suggesting that the high dose of EBN used in this study was effective in preventing hypercholesterolemia. Simvastatin is used to manage hypercholesterolemia, and the present results demonstrate its effectiveness [12]. However, the results from this study also suggest that EBN may be as effective as simvastatin in preventing hypercholesterolemia, possibly because it contains multiple bioactive compounds that can regulate different processes [13]. There was a significant increase in triglycerides level of the HFD group compared to that of the control group. This effect was ameliorated by the administration of both low and high doses of EBN as similarly observed with simvastatin. In addition, elevated levels of LDL are a known risk factor for cardiovascular diseases [14, 15]. However, as opposed to simvastatin, a high dose of EBN significantly reduced the elevated LDL levels observed in the HFD group. Thus, EBN plays a potential role in preventing cardiovascular diseases.

### 3.3. Liver Enzymes, Urea, and Creatinine

Serum alanine transaminase (ALT), aspartate transaminase (AST), alkaline phosphatase (ALP), and lactate dehydrogenase (LDH) are important liver enzymes that are used clinically to determine the health status of the liver [16]. Normally, liver enzyme levels remain within a normal range in the absence of damage in the liver. In the presence of a toxic factor, they become deranged [17]. Hyperlipidemia has been associated with elevated liver enzymes due to fatty liver deposits [18]. In this study, the liver enzyme levels were significantly different between the normal and HFD groups (Figure 1), suggesting that hyperlipidemia which was induced by HFD caused liver damage. Although simvastatin is effective in managing hypercholesterolemia, it could not ameliorate the negative effects of HFD on liver function enzymes. This is demonstrated by the elevated enzyme levels in the present study. EBN groups, on the other hand, attenuated the HFD-induced deterioration of liver enzymes, significantly better than the HFD and HFD + SIM groups.

Similarly, EBN attenuated HFD-induced kidney damage (Figure 2). The kidneys play an important role in removing metabolic wastes from the body, and they are common targets of toxic damage. Studies have demonstrated that hyperlipidemia often leads to kidney damage [19] similar to what was observed in the HFD group. Higher serum lipid levels may have increased the viscosity of blood in the HFD group leading to reduced blood flow to the kidneys. The kidneys are sensitive to the reduced blood flow volume and, as such, may have resulted in increased urea and uric acid levels. The improved urea and uric acid levels in the EBN and simvastatin groups may also have been a result of the improved lipid profiles and subsequently reduced blood viscosity [20, 21].

### 3.4. Lipase Activity

Lipase is an esterase enzyme that catalyzes the hydrolysis of lipids and plays an important role in the digestion, transport, and processing of dietary lipids [22]. Increased lipase activity is most commonly associated with pancreatitis [22]. This study showed a significant decrease in the level of triglycerides in the EBN groups compared to that of the HFD group. Moreover, coupled with the increased triglycerides levels in the HFD group, elevated levels of lipase activity may also indicate lipid abnormalities as seen in the present study.  Figure 3 shows the results of the lipase activity. The HFD group had a higher level than the normal and HFD + EBNH groups. The reason may be due to the higher level of lipids which increased the burden on the pancreas, thus stimulating the release of more lipase. Moreover, this can also be explained by the documented links between hypertriglyceridemia and pancreatitis [23].

### 3.5. OxLDL

OxLDL is produced from the oxidative modification of LDL and has been shown to cause more damage than LDL. OxLDL has been demonstrated to play a key role in the development of atherosclerosis, and its circulating concentrations have been shown to reflect the state of pathological atherosclerosis and the risk of coronary artery disease [24].  Figure 4 shows that the HFD group had a significantly higher oxLDL level than normal and HFD + EBNH groups. This suggests a high risk of CVD in the HFD group, which can be attenuated by EBN.

### 3.6. Histological Analyses

Fatty liver is often seen in hyperlipidemia, as seen in the HFD group in the present study (Figure 5). The histological data corroborate the hypercholesterolemia in the HFD and the worsened liver enzymes. Conversely, the EBN group had fewer fatty deposits in the liver confirming the effectiveness of EBN in attenuating HFD-induced lipid abnormalities.

### 3.7. Hepatic mRNA Levels of Lipid Metabolism Genes

The HFD group worsened the transcriptional regulation of cholesterol-related genes, which were attenuated by EBN (Figure 6). These transcriptional changes possibly underlie the lipid profile changes observed in the groups. HFD feeding downregulated the expressions of LDLR and CYP7A1 genes, which are involved in the mediation of endocytosis of cholesterol-rich LDL and cholesterol synthesis, respectively. Moreover, low LDLR levels have been associated with high serum cholesterol levels due to reduced LDL clearance and have been linked to the progression of atherosclerosis [25], while upregulation of CYP7A1 contributes to increased bile acids production and reduced cholesterol levels [26]. Furthermore, HFD feeding upregulated the PCSK9, APOB, and HMGCR genes, which are key cholesterol metabolism genes. PCSK9 regulates cholesterol homeostasis by inducing LDLR degradation [27, 28], which may then prevent the clearance of LDL from the blood and eventually lead to hypercholesterolemia [28]. HMGCR, on the other hand, is the rate-limiting enzyme in cholesterol synthesis through the mevalonate metabolic pathway, whose expression is closely regulated with that of LDLR. HMGCR activity can be suppressed by cholesterol synthesis, leading to an increased hepatic LDLR expression. ApoB is the primary apolipoprotein of LDL, IDL, VLDL, and chylomicrons, which is responsible for transporting lipids from the liver to the cells. Increased ApoB levels have been associated with higher concentrations of LDL and an increased risk of CVD [29] and insulin resistance [30]. Overall, the HFD-induced lipid perturbations were regulated by EBN similar to simvastatin indicating that EBN was effective in regulating hepatic cholesterol metabolism.

## 4. Conclusions

In the present study, we have demonstrated that HFD-induced hypercholesterolemia worsened liver and kidney functions, partly through dysregulation of hepatic cholesterol metabolism. EBN, on the other hand, attenuated HFD-induced lipid perturbations partly via transcriptional regulation of cholesterol metabolism genes as against simvastatin used to manage hypercholesterolemia which could have acted through a different mechanism. EBN can, therefore, be used as a supplement to lower the risk of CVD due to lipid abnormalities.

## Figures and Tables

**Figure 1:** Serum alanine transaminase (ALT), aspartate transaminase (AST), alkaline phosphatase (ALP), and lactate dehydrogenase (LDH) in high-cholesterol diet-fed rats after 12 weeks of intervention. Bars with different letters in each panel indicate a statistical difference (*p* < 0.05).

**Figure 2:** Serum urea, creatinine, and uric acid in high-cholesterol diet-fed rats after 12 weeks of intervention. Bars with different letters in each panel indicate a statistical difference (*p* < 0.05).

**Figure 3:** Serum lipase in high-cholesterol diet-fed rats after 12 weeks of intervention. Bars with different letters in each panel indicate statistical difference (*p* < 0.05).

**Figure 4:** Serum oxLDL in high-cholesterol diet-fed rats after 12 weeks of intervention. Bars with different letters in each panel indicate statistical difference (*p* < 0.05).

**Figure 5:** The histological changes in the liver of different groups.

**Figure 6:** Effects of EBN on hepatic tissue mRNA levels of PCSK9, Apob, CYP7A1, HMGR, and LDLR in HFD-fed rats. Bars with different letters in each panel indicate statistical difference (*p* < 0.05).

**Table 1:** Names and primer sequences used in the study.

Name	Left sequence	Right sequence
B2m^a^	AGGTGACACTATAGAATAATGCTTGCAGAGTTAAACA	GTACGACTCACTATAGGGATGCATAAAATATTTAAGGTAAGA
Hprt1^a,b^	AGGTGACACTATAGAATATCCTCATGGACTGATTATG	GTACGACTCACTATAGGGACTGGTCATTACAGTAGCTCTT
Rpl13a^a^	AGGTGACACTATAGAATAATGGGATCCCTCCAC	GTACGACTCACTATAGGGAATTTTCTTCTCCACATTCTT
Kan(r)^c^		
CYP7A1	AGGTGACACTATAGAATAATAACATCCGAAAAGATGAC	GTACGACTCACTATAGGGATTTCCATTACTGTAGAAGGTG
LDLR	AGGTGACACTATAGAATAATGAGGTACGTAAGATGACC	GTACGACTCACTATAGGGAAGGTCAGACCAGTAAATTCT
PCSK9	AGGTGACACTATAGAATATGATTAATGCAGATCAGTTC	GTACGACTCACTATAGGGATTTATGTCCTAGCATCACTG
ApoB	AGGTGACACTATAGAATAATATCCTGAACATCAAGAGG	GTACGACTCACTATAGGGAGATGCTGTTCATTACAGATG
HMGCR	AGGTGACACTATAGAATATCATTCATTTCCTCGACA	GTACGACTCACTATAGGGATCTCCCTTACTTCATCCTGT

^a^Housekeeping genes. ^b^Normalization gene. Underlined sequences are universal left and right sequences (tags). ^c^Internal control was supplied by Beckman Coulter Inc (Miami, FL, USA) as part of the GeXP kit. RT conditions were as follows: 48°C for 1 min, 37°C for 5 min, 42°C for 60 min, 95°C for 5 min, and then maintained at 4°C. PCR conditions were initial denaturation at 95°C for 10 min, followed by two-step cycles of 94°C for 30 s and 55°C for 30 s, ending in a single extension cycle of 68°C for 1 min. B2m: beta-2-microglobulin; Hprt1: hypoxanthine phosphoribosyltransferase 1; KanR: kanamycin resistant; Rpl13a: ribosomal protein L13a; CYP7A1: cholesterol 7 alpha-hydroxylase; LDLR: low-density lipoprotein receptor; PCSK9: proprotein convertase subtilisin/kexin type 9; ApoB: apolipoprotein B; HMGCR: HMG-CoA reductase/3-hydroxy-3-methyl-glutaryl-CoA reductase.

**Table 2:** Food composition, food intake, body weight, and lipid profile.

Animal group	Component ratio (%)	Additional component (%)	Food intake (Kcal/kg/day)	Initial weight (g)	Final weight (g)	Chol. (mmol/L)	Trig. (mmol/L)	LDL (mmol/L)	HDL (mmol/L)	LDL/HDL	TG/HDL
Normal	100 : 0 : 0 : 0	0	215.5 ± 33.5^a^	260.4 ± 10.7^a^	384.0 ± 22.9^a^	1.55 ± 0.43^a^	0.62 ± 0.15^a^	0.28 ± 0.11^a^	1.18 ± 0.35^a^	0.24 ± 0.04^a^	0.55 ± 0.15^a^
HFD	65 : 5 : 20 : 10	0	215.0 ± 37.5^a^	262.6 ± 17.7^a^	395.2 ± 16.8^a^	7.47 ± 1.13^b^	1.21 ± 0.38^b^	4.98 ± 1.03^b^	1.05 ± 0.13^a^	4.77 ± 0.98^b^	1.16 ± 0.33^b^
HFD + SIM	65 : 5 : 20 : 10	Simvastatin (10 mg/kg)	215.7 ± 36.6^a^	267.7 ± 21^a^	375.7 ± 53.4^a^	4.99 ± 1.11^c,d^	0.63 ± 0.18^a^	3.60 ± 1.1^b,c^	1.04 ± 0.17^a^	3.46 ± 0.94^b,c^	0.62 ± 0.22^a,b^
HFD + EBNL	62.5 : 5 : 20 : 10	2.5% EBN	216.1 ± 36.8^a^	261.7 ± 15.4^a^	380.7 ± 25.6^a^	6.04 ± 0.75^b,c^	0.54 ± 0.1^a^	4.52 ± 0.71^b,c^	1.17 ± 0.18^a^	3.94 ± 0.88^b,c^	0.46 ± 0.08^a^
HFD + EBNH	45 : 5 : 20 : 10	20% EBN	216.5 ± 35.8^a^	257 ± 20.1^a^	368.0 ± 29.3^a^	4.17 ± 1.06^d^	0.44 ± 0.1^a^	2.98 ± 0.83^c^	1.18 ± 0.29^a^	2.63 ± 0.87^c^	0.38 ± 0.08^a^

EBN: edible bird's nest. Component ratio: normal pellet% : cholesterol : palm oil : starch. Columns with different letters indicate statistical difference (*p* < 0.05).

## Data Availability

Data are available from corresponding authors upon request.

## Abbreviations

ALP: Alkaline phosphatase
ALT: Alanine transaminase
ApoB: Apolipoprotein B
AST: Aspartate transaminase
CYP7A1: Cholesterol 7 alpha-hydroxylase
EBN: Edible bird's nest
EBNL: Low dose of edible bird's nest
EBNH: High dose of edible bird's nest
HDL: High-density lipoprotein
HFD: High-cholesterol diet
HMGCR: HMG-CoA reductase/3-hydroxy-3-methyl-glutaryl-CoA reductase
LDH: Lactate dehydrogenase
LDL: Low-density lipoprotein
LDLR: Low-density lipoprotein receptor
oxLDL: Oxidized low-density lipoprotein
PCSK9: Proprotein convertase subtilisin/kexin type 9
TC: Total cholesterol
TG: Triacylglycerol.
